The article "Fluorescent Carbon Dot-Supported Imaging-Based Biomedicine: A Comprehensive Review" was retracted in 2023. Reasons: signs of a paper mill; compromised peer review; unreliable results or conclusions.

# Fluorescent Carbon Dot-Supported Imaging-Based Biomedicine: A Comprehensive Review

**DOI:** 10.1155/2022/9303703

**Published:** 2022-04-10

**Authors:** Le Minh Tu Phan, Sungbo Cho

**Affiliations:** ^1^School of Medicine and Pharmacy, The University of Danang, Danang 550000, Vietnam; ^2^Department of Electronic Engineering, Gachon University, Seongnam, Gyeonggi-do 13120, Republic of Korea; ^3^Department of Health Sciences and Technology, GAIHST, Gachon University, Incheon 21999, Republic of Korea

## Abstract

Carbon dots (CDs) provide distinctive advantages of strong fluorescence, good photostability, high water solubility, and outstanding biocompatibility, and thus are widely exploited as potential imaging agents for *in vitro* and *in vivo* bioimaging. Imaging is absolutely necessary when discovering the structure and function of cells, detecting biomarkers in diagnosis, tracking the progress of ongoing disease, treating various tumors, and monitoring therapeutic efficacy, making it an important approach in modern biomedicine. Numerous investigations of CDs have been intensively studied for utilization in bioimaging-supported medical sciences. However, there is still no article highlighting the potential importance of CD-based bioimaging to support various biomedical applications. Herein, we summarize the development of CDs as fluorescence (FL) nanoprobes with different FL colors for potential bioimaging-based applications in living cells, tissue, and organisms, including the bioimaging of various cell types and targets, bioimaging-supported sensing of metal ions and biomolecules, and FL imaging-guided tumor therapy. Current CD-based microscopic techniques and their advantages are also highlighted. This review discusses the significance of advanced CD-supported imaging-based *in vitro* and *in vivo* investigations, suggests the potential of CD-based imaging for biomedicine, and encourages the effective selection and development of superior probes and platforms for further biomedical applications.

## 1. Introduction

Bioimaging plays a significant role in understanding the structure and biological processes of biomolecules, living cells, tissues, organs, and organisms [1]. Imaging has rapidly become an essential approach in biomedical applications due to its possibility to improve the prevention, detection, and treatment of disease. The powerful bioimaging techniques of fluorescence microscopy (FM) make it a prerequisite for taking advantage of many medical applications in preclinical studies and clinical interventions, by providing excellent imaging of anatomical structures and molecular imaging of specific biomarkers, as well as functional imaging of physiological activities [2, 3]. Compared to small fluorescent molecules (rhodamine, fluorescein,…) or semiconductor quantum dots, highly fluorescent (FL) carbon dots (CDs) that exhibit more advanced properties are currently being developed for various applications owing to their unique properties, such as multicolor emissions, excellent photostability and biocompatibility, and easy surface functionalization [4]. They can be easily synthesized in a one-step process using microwave or hydrothermal methods with environmental friendliness and affordability. With non-toxicity, high water solubility, strong fluorescence, and two-photon excitation (TPE) capability, CDs are broadly utilized in live-cell imaging, catalysis, electronics, biosensing, targeted drug delivery, and imaging-guided biomedical applications [5]. Taking advantage of the strong fluorescence of CDs has accelerated the intensive investigation of the biomedical sciences, especially in bioimaging-supported fields, providing significant benefits in effective bioimaging-supported medicine. The combination between CDs and advanced imaging technologies might increase the precision and accuracy of biomedical applications.

Various reports in the literature have summarized the synthesis, properties, and applications of CDs, in the biosensing and theragnostic fields [5–8] to emphasize the applicable potential of CDs for biomedical applications. These reviews broadly discussed the applications of CDs including bioimaging, sensing, and therapy, without deeply focusing on bioimaging-based medicine. Imaging in modern biomedicine is especially beneficial procedure in the interest of diagnosing, monitoring, or treating disease, making it extremely significant in medical fields. Therefore, an overview of bioimaging-supported biomedical sciences that focuses on the excellent bioimaging properties of CDs is needed to explore the potential significance of CDs in the field of imaging-supported medical applications. Hence, this review emphasizes the exploitation of current CD-based FL imaging as powerful nanoprobes for advanced biomedical applications that include pristine bioimaging, bioimaging-supported sensing platforms, and bioimaging-guided therapy. The carbon dot-supported microscopic techniques are highlighted, along with their advantages for effective bioimaging purposes. The latest research on the CD-based bioimaging-supported biomedical applications is also comprehensively reviewed. In particular, the imaging of different species targets (cells, organelles, bacteria, fungi, animals), the monitoring of various metal ions and biomolecules in live cells and tissue, and the imaging-guided therapeutics of tumors (Figure 1). This review provides an interesting focus on advanced innovation for further *in vitro* and *in vivo* investigation based on bioimaging to develop superior platforms for efficient healthcare study. The challenges and perspectives are also discussed for considering the future of these CD-supported imaging-based biomedical sciences.

## 2. Current Carbon Dot-Supported Microscopic Techniques

Microscopic imaging has paved the way for a revolution as a major technique for the visualization and understanding of the structure and physiology of cells and tissues that provides unprecedented insights into the biological processes related to physiological and disease processes, as well as supports various biomedical applications [9, 10]. There are two types of FM techniques that can or cannot overcome the resolution limit where the objects become unresolvable if the distance between the two-point objects is less than half of the wavelength of the excitation source, namely the diffraction-limited and super-resolution microscopy techniques, respectively. Diffraction-limited microscopy techniques consist of epifluorescence illumination microscopy, confocal laser scanning microscopy (CLSM), total internal reflection FM, and light-sheet FM, while super-resolution microscopy techniques include photoactivated localization microscopy, stochastic optical reconstruction microscopy, and ground-state depletion, followed by individual return microscopy, stimulated emission by depletion microscopy, structured illumination microscopy, binding-activation localization microscopy, and scanning near-field optical microscopy. Microscopic techniques are optimally selected depending on the spatial organization of the biological entity, temporal dynamics, and susceptibility to phototoxicity [11, 12]. For specific CD-supported microscopic techniques, scientists have mainly focused on the use of optical and electron microscopy techniques that include FM, CLSM, and single-photon and two-photon excitation microscopy for *in vitro* studies, and *in vivo* fluorescence imaging systems for *in vivo* studies, as shown in Table 1, which techniques are mainly applied in the fields of cell biology or biomedical sciences [115]. These FM techniques have been widely exploited using FL CDs for biomedical applications that include the imaging of cells and tissues, imaging-based sensing *in vitro* and *in vivo*, and imaging-guided therapy. CLSM obtains superior quality of FL images by improving the signal-to-noise ratio compared to widefield microscopy, two-photon excitation microscopy enables imagery of high depths, which is unachievable by single-photon excitation microscopy [94, 116–118]. Taking advantage of CDs, the CD-supported FM has been successfully exploited as an ideal candidate for diverse biomedical applications, such as providing active physiological processes through the imaging of species in live cells or tissues, as well as support for therapeutic applications to disease.

## 3. Fluorescent Carbon Dots for Bioimaging Applications

Table 1 summarizes the latest research of various CDs based on the precursors of synthesis, applied color, and excitation/emission wavelengths for bioimaging of various targets such as cells, organelles, bacteria, fungi, and animal models. Case studies of CD-based bioimaging are then discussed in this section, according to biotarget.

### 3.1. Fluorescent Carbon Dots for the Bioimaging of Cells and Tissues

Various multicolor FL CDs have been widely fabricated and applied as excellent nanoprobes to effectively image cells and tissues. By simply mixing glucose as a carbon source, EDA as an N-dopant, and phosphoric acid as P-dopant, water-soluble FL nitrogen and phosphorus dual-doped carbon dots (NP-Cdots) of about 3.5 nm in diameter were rapidly synthesized by the acid-base neutralization spontaneous heat, and they exhibited multicolor fluorescence, with the optimal excitation and emission wavelengths at (403 and 502) nm, respectively. These biocompatible NP-Cdots were utilized as a multicolor FL agent for the intracellular imaging of human cervical carcinoma SiHa cells. The multicolor fluorescence of cells stained with NP-Cdots presented blue, green, yellow, and red Em under laser stimulation at 405, 488, 515, and 543 nm, respectively, showing internalization and good decentralization into the cytoplasm of SiHa cells, along with the entering of some NP-Cdots into the cell nucleolus. These results indicate the excellent ability of these NP-Cdots to permeate the cell membrane for the application in *in vitro* cellular imaging (Figure 2(a)) [25]. The double rare-earth-doped (gadolinium, ytterbium) carbon dots (Gd/Yb@CDs) of 5.26 nm in diameter were fabricated via a one-step hydrothermal process at 200°C for 10 h using Na_2_EDTA and L-arginine as raw materials, and GdCl_3_ and YbCl_3_ as dopants. These Gd/Yb@CDs exhibited Ex-dependent Em, with the strongest Em at 418 nm when excited at 340 nm, superhigh photostability without change of fluorescence intensity for 2 h, and superior biocompatibility without toxicity to HeLa cells up to 1 mg/mL of Gd/Yb@CDs. The *in vitro* HeLa cells and *in vivo* nude mice treated with Gd/Yb@CDs displayed significant blue fluorescence with very weak interference from the autofluorescence of cells [73].

Various o-, m-, or p-phenylenediamines (pDA) with triethylenetetramine as precursors were used to synthesize the FL carbon dots with different colors for the imaging application of cellular ribonucleic acids (RNA). However, only m-phenylenediamines formed carbon dots (m-CDs) with a size of 2.75 nm, and maximum green Em at 510 nm under Ex at 360 nm demonstrated excellent ability to specifically bind to the cellular RNA of HEp-2 cells, allowing successful long-term real-time monitoring of RNA dynamics during cell apoptosis, mitosis, and proliferation. The RNA affinity of m-CDs is associated with the isoquinoline moieties and amines on the surface of m-CDs that bind to RNA through *π*–*π* stacking and electrostatic bonding, respectively. Furthermore, investigations of the *in vivo* zebrafish larvae body showed major accumulation in the lens, pronephros, intestine, and vessels, suggesting the efficient excretion of m-CDs after 48 h of incubation. Hence, m-CDs as smart nanoprobes for cellular RNA imaging could be valuable for the development of visualized screening of RNA [60]. Interestingly, hydrogen-bonding-induced Em CDs (HBIE-CDs) formed by a hydrothermal method using m-phenylenediamine (mDA) and folic acid (FA) as precursors displayed 460 nm of blue Em in nonhydrogen-bonding solution and 535 nm of green Em in hydrogen-bonding solution due to the inhibition of nonirradiation by a H-bond network. The HBIE-CDs possessed strong affinity toward nucleic acid as the donor of H-bond without interference, dramatically increasing 6-fold green fluorescence after binding with the DNA or RNA of Hela cells. After incubation of Hela cells with HBIE-CDs for 5 min, cells without washing exhibited strong green fluorescence in the nucleus after binding with DNA and RNA and almost no background fluorescence in the cytoplasm, which was almost similar to cells with PBS washing, allowing continuous monitoring of the cell nucleus without interruption (Figure 2(b)) [61]. Furthermore, monitoring the dynamics of DNA and RNA structures in live cells is essential for tracking cell behavior. However, the difficulty in fabricating a the nanoprobe that can distinguish between double-stranded DNA and single-stranded RNA, and cross multiple membrane barriers from the cell to the tissue level is still a challenge. Thus, a cationic carbon quantum dot of 2–3 nm in diameter and zeta potential at +20 mV synthesized from conductive carbon nanoparticles and p-phenylenediamine was successfully developed to address this challenge. The CD exhibited green fluorescence at 510 nm under 400 nm Ex, but significant fluorescence enhancement was obtained with the existence of DNA, up to 8-fold, due to the CD insertion into the grooves of dsDNA that restricted the rotation of the linkage bonds between the pDA and the CD core. In contrast to DNA, the presence of RNA induces the shift of Em fluorescence to red at around 620 nm under 540 nm Ex, because it leads to the formation of CD aggregates to make the strong fluorescent transit from green to red. Upon treatment of CD, the nuclei of a total of 12 cell types emitted strong green fluorescence under 488 nm Ex, while strong red fluorescence was observed in the cytoplasm under 542 nm Ex, due to the CD staining of DNA and RNA, respectively, indicating its ability to cross both the plasma and nuclear membranes to dye the target DNA and RNA. The CD's ability to enter the intestinal pathway was confirmed through the greater concentration of CD in intestinal wall cells using the imaging of wireworms. Further, it was successfully applied to monitor DNA and RNA during cell division at different cell cycles, including prophase, metaphase, telophase, and interphase. CD's selectivity towards DNA and RNA, and the excellent ability to penetrate through various biological barriers in cells and live organisms, make CD an efficient agent for basic cell biology, embryology, and clinical diagnosis [104].

Lysosomes, as another subcellular organelle, also play critical roles in protein degradation, cell signal transduction, plasma membrane repair, homeostasis, and autophagy, making the development of a specific probe for the imaging of lysosomes extremely necessary to understand the dysfunction of lysosomes that is related to various diseases, such as Alzheimer's disease, neurodegenerative diseases, and cancer. Through the conjugation of the morpholine group (ML) as lysosome targeting to CDs formed from polyethyleneimine (PEI) and citric acid (CA) as precursors, CDs-PEI-ML were successfully fabricated to act as a long-term tracking probe of lysosomes for cell imaging with excellent properties that include strong blue Em, high photostability, adequate biocompatibility, and high selectivity toward lysosomes. Imaging of the lysosomal localization of CDs-PEI-ML in live Hela cells was described that CDs-PEI-ML were translocated into lysosomes via an endocytic pathway, and accumulated in acidic lysosomes with less diffusion into the cytoplasm due to the presence of lysosome target group morpholine on the surface of CDs-PEI-ML. This CDs-PEI-ML exhibited high specificity in lysosomal imaging, presenting an alternative FL probe for lysosome labeling and imaging (Figure 2(c)) [70].

Mitochondrion as a vital energy-supplying organelle, plays an important role in cellular functions, such as the generation of ATP and reactive oxygen species (ROS), regulation of transmembrane potentials, and initiation of apoptosis and autophagy, making the dysfunction of the mitochondrial responsible for various diseases, such as Alzheimer's disease, Parkinson's disease, diabetes, and cancer. The green FL CDs synthesized using chitosan, ethylenediamine, and mercaptosuccinic acid as precursors, showed intrinsic mitochondrial targeting ability to visualize mitochondria for bioimaging. These CDs quickly entered cells and specifically targeted mitochondria through energy-dependent, caveolae-mediated endocytosis, exhibiting superior features that included multicolor fluorescence, good photostability, and long-term imaging capability for at least 24 h, compared to MitoTrackers (commercial mitochondrial probes), representing a good FL nanoprobe for mitochondrial imaging that could be an alternative to commercial probes (Figure 2(d)) [63].

As another targeting species in cellular bioimaging, hyaluronan (HA), a linear long-chain polymer, is intimately associated with human tumor progression by stimulating growth, survival, and angiogenesis within primary tumors or their metastases. About 3.2 nm N-doped CDs using starch as a carbon source and L-tryptophan as nitrogen dopants were coupled with molecularly imprinted polymer (MIP) and glucuronic acid (GlcA) as an epitope of hyaluronan to form CD-MIPGlcA that was employed to probe HA cancer biomarkers. CD-MIPGlcA with (3–10) nm diameter emitted the green maximum Em at 500 nm under 445 nm Ex with high selectivity to HA, showing about 4 times higher FL intensity on HeLa cells than that on HaCaT cells, suggesting the ability of CD-MIPGlcA to differentiate between cancer cells and normal cells. The possibility of CD-MIPGlcA in HA-targeting FL nanoprobes indicates how powerful these tools are for the imaging of tumor biomarkers [71].

A desirable goal in bioimaging applications is to discriminate against interference from autofluorescence. However, it is still a challenge to develop room temperature (RT) phosphorescence (RTP) probes that feature ultralong Em lifetimes. CD-based silica composites (CDs@SiO_2_) with long Em lifetimes of 1.64 s were successfully fabricated for ultralong lifetime phosphorescence imaging of cells and tissue at RT using polyacrylic acid and EDA as CD precursors. CDs@SiO_2_ emitted blue fluorescence and the afterglow green Em maximum at 520 nm under an Ex of 356 nm. Although due to strong endogenous autofluorescence at 365 nm irradiation, it was difficult to distinguish between CDs@SiO_2_-untreated and treated onion bulb epidermal tissues, strong green phosphorescence of the CDs@SiO_2_-treated group in EM-6 mouse breast carcinoma cells and onion bulb epidermal tissue was observed after turning off the irradiation, highlighting the successful phosphorescence imaging of CDs@SiO_2_ in bioimaging in cells or plant and animal tissues by eliminating the autofluorescence interference. These CDs@SiO_2_ could serve as excellent nanoprobes for bioimaging with an efficient ability to discriminate against tissue autofluorescence, suggesting the potential for ultralong-lived RTP reporters [64]. In addition, a CD-grafted cellulose hybrid phosphor with a high affinity to bind cellulose was prepared for effective fluorescence mapping of cellulosic plant cell walls. These reddish-orange emissive CDs exhibited strong fluorescence at 633 nm with a 44% high quantum yield and high photostability. Various model plant tissues, including onion bulb epidermal tissue, the root of mung bean sprout, and the stem and leaf of *Arabidopsis thaliana*, were employed to demonstrate the bioimaging capacity of these CDs. CDs can readily have absorbed in plant tissues and bind to a cellulose-rich structure with deep penetration to 55.5 *μ*m depth in the stem of *Arabidopsis thaliana*, 177.2 *μ*m in the root of mung bean sprout, and 136.3 *μ*m in onion bulb epidermal tissue, respectively, which could address the limitation of FL dyes in their difficulty in visualizing deeper tissue layers of ≥ (50 to 100) *μ*m. These CDs could serve as useful probes for the study of cell wall structure in living plant cells (Figure 2(e)) [81].

Undoubtedly, CDs exhibit excellent performance for bioimaging applications that can enhance the understanding of cells or tissues. CDs can also be applied as nanoprobes for the recognition of cancerous cells from normal cells. However, each specific mechanism of interaction between CDs and targets in cells or tissues, cytotoxicity, and optimal conditions of bioimaging processes should be carefully studied to contribute significantly to biological and biomedical sciences.

### 3.2. Fluorescent Carbon Dots for the Bioimaging of Bacteria

Bacteria are abundant in the natural world and can lead to global bacterial infection, so it is essential to accurately specify them for efficient treatment. Nitrogen and sulfur codoped CDs (NSCDs) were obtained by a microwave-assisted hydrothermal method using thiourea as a precursor in tris-acetate-ethylenediamine (TAE) buffer, for use in the imaging of various bacteria. These NSCDs were well mono-dispersed with an average size of 3.62 nm and exhibited maximum fluorescence at 426 nm Em under irradiation of 340 nm with a quantum yield of 57%. With no toxicity to bacteria cells, NSCDs internalization or endocytosis occurred after incubation with bacteria, and emitted blue fluorescence that was observed in *E. coli, Pseudomonas*, and *Staphylococcus*, but not in *Klebsiella.* The untagging effect on *Klebsiella* may have resulted in the decimation or disorientation of NSCDs due to the catabolic characteristic of *Klebsiella* for different aromatic compounds. Additionally, the multicolor fluorescence of NSCDs as imaging nanoprobes was screened under different Ex wavelengths of (380, 450, and 505) nm in tagged *E. coli* cells, showing the bright colors of blue, green, and red at (430, 525, and 590) nm Ems, respectively [20].

Taking advantage of the selective binding affinity of boronic acid to diols groups on the bacterial cell wall, phenylboronic acid-functionalized FL carbon dots (FCDs) with strong blue fluorescence were synthesized and conjugated to dye molecules, then successfully applied in the selective detection of bacteria via the imaging of diol-containing bacteria. Owing to the preferential affinity of phenylboronic acid toward diol-containing molecules through cyclic ester bond formation, glucose-containing bacteria were replaced with dye molecules that led to the release of dye from the FCD to recover the fluorescence, gradually increasing the FL intensity from (0 to 60) min under 405 nm Ex in the presence of *E. coli* or *S. aureus.* These FCDs exhibited high sensitivity and chemical specificity for bacteria detection via fluorescence imaging (Figure 2(f)) [15].

Accurate bacterial identification is required to characterize unknown bacteria, which is important for the fast diagnosis of bacterial infections. A one-pot solvothermal approach was exploited to obtain a quaternized CDs using glycerol and dimethyloctadecyl[3-(trimethoxysilyl)propy] ammonium chloride (Si-QAC) for the identification of gram-type bacteria through bacteria imaging. Si-QAC containing CDs interacted with the negatively charged bacterial cells via both electrostatic and hydrophobic interactions, selectively connecting with the gram-positive bacteria due to the different surfaces of gram-positive and gram-negative bacteria. CDs displayed Ex-dependent fluorescence from (320 to 500) nm with maximum intensity at 473 nm under 360 nm Ex, significantly enhancing the blue fluorescence once the CDs are adsorbed onto the *S. aureus* gram-positive bacteria, but not the *E. coli* cells, in the mixture of these bacteria. This CD-based Gram-type differentiation method was accurate, fast, and facile, suggesting that this CD FL staining method could act as an alternative to the conventional gram staining method for differentiating gram-type bacteria (Figure 2(g)) [14].

CD-based bioimaging of bacteria is successfully utilized for FL imaging or differentiating gram-type bacteria. Nevertheless, these studies mostly focused on the imaging of several bacteria, such as *S. aureus,* and *E. coli,* other bacterial types that possess different influences should be further investigated. A CD with specific affinity towards each bacterium should be developed for efficient application. Cytotoxicity of CDs should be considered carefully for various types of bacteria for further utilization. The interference of culture media to FL of CDs and the real-time ability of monitoring bacteria are required to study deliberately.

### 3.3. Fluorescent Carbon Dots for the Bioimaging of Fungi

Along with bacteria, the bioimaging of fungi is also important to understand the fungal biology or their infection mechanisms more clearly. Carbon dots synthesized from methyl red (MR) as a precursor in the presence of ethylenediamine (EDA) by facile hydrothermal pyrolysis, namely as MR-EDA-CDs, were fractionated into four fractions with different sizes of (16.3, 12.6, 5.5, and 4.5) nm under column chromatography that emitted green, purple, blue, and yellow fluorescence at (398, 470, 511, and 530) nm, respectively. These biocompatible MR-EDA-CDs were investigated as imaging nanoprobes for the FL imaging of pathogenic fungal cells (*C. gloeosporioides*). MR-EDA-CDs internalized into the fungal cells upon 6 h of incubation at RT, brightly illuminating the multicolor fluorescence with Ex at 405 nm by confocal microscopy (Figure 2(h)) [99].

Owing to their ease of availability and affordability, natural resources have been widely used as precursors for the preparation of CDs. *Acacia concinna* fruit seeds (shikakai) as a green precursor were used to fabricate CDs in the application as biocompatible nanoprobes for the multicolor imaging of fungal (*Penicillium* sp.) cells. Upon Ex of 390 nm, these CDs displayed a strong Em peak at 468 nm with a higher quantum yield (10.2%), with good biocompatibility with fungal cells. The ultra-small CDs (2.5 nm diameter) internalized into the cells via endocytosis, and located in the cytoplasm and especially the nucleus of cells, exhibiting bright blue, green, and red fluorescence colors under laser Ex wavelengths of (405, 488, and 561) nm [100]. Another multicolor emissive CD that generated blue, green, and yellow fluorescence was obtained from *Manilkara zapota* fruits in acidic solutions (sulphuric acid and phosphoric acids) at different temperatures of 100 and 80 °C for 60–15 min. These CDs exhibited the maximum Em peaks at 443, 515, and 563 nm (blue, green, and yellow) under excitation at 350, 420, and 440 nm, with the QYs of 5.7, 7.9, and 5.2 %, respectively. Due to the small size of these CDs of from 1.9–4.5 nm, they are easily internalized into *Aspergillus aculeatus* and *Fomitopsis* sp. cells via the cell membrane through endocytosis, located in the cell membrane and cytoplasm, resulting in blue, green, and yellow fluorescence at Ex wavelengths of 405, 488, and 561 nm with good intensity [101]. Overall, the FL CDs have proven to be potential agents for the multicolor imaging applications of fungal cells. However, there are many other types of fungi that are essential to be explored as well. These reported CDs are mainly for imaging of the whole bodies of fungi. Specific CDs for different organelles in fungi are thus highly required to develop for obvious understanding.

### 3.4. Fluorescent Carbon Dots for the Bioimaging of Animal Models

*In vivo* molecular imaging as a powerful tool for the analysis of the body significantly contributes to precise medicine through diagnosis and guiding therapy. N-doped carbon dots (NCDs) obtained by a hydrothermal method using pDA as precursor have embedded with Mn2+ onto the polydopamine (PDA) nanoparticle (NP) to fabricate the imaging nanoprobe, namely as PDA@NCDs(Mn). Using NCDs as FL agents, PDA as a photothermal agent, and Mn^2+^ as a T2 magnetic resonance contrast agent, these CD-based NPs were successfully applied as multimodal imaging nanoprobes for tumor diagnosis. These PDA@NCDs(Mn) NPs displayed maximum Em peak at 620 nm when Ex at 550, with strong red Em under the Ex wavelength of 500 nm. For *in vivo* fluorescence imaging investigation, PDA@NCDs(Mn) were injected into the left rear flank region of the mice model, then accumulated in the tumor site with good distribution, hence valid fluorescence was observed around the tumor. After 12 h post-injection, organs (heart, liver, spleen, lung, and kidney) and tumors were harvested to assess fluorescence intensities. These PDA@NCDs(Mn) NPs mainly accumulated in the liver, lung, and kidney tissues, as well as stronger fluorescence signal in tumor tissues than the spleen and heart, which was observed in a time-dependent fluorescence intensity manner, indicating red-emissive PDA@NCDs(Mn) NPs as promising fluorescence imaging agent for *in vivo* imaging (Figure 3(a)) [107]. Phosphonated compounds are widely applied for the imaging and treatment of severe bone turnover due to their high affinity to hydroxyapatite (HA) minerals. monophosphonated CDs obtained by a one-pot hydrothermal method using food-grade agave nectar and *α*-methoxy-*ω*-phosphate polyethylene glycol exhibited Ex-dependent Em spectra with maximum Ex/Em at 430/600 nm and high affinity towards calcium salt of the bone, indicating their potential as bone-seeking luminescent nanoprobes for the detection of bone microcracks via fluorescence imaging. The CDs-injected mice displayed a prominent difference in the luminescent emitted from the tibia when excited at 430 nm and imaged at 600 nm, suggesting that CDs can light up the tissue surrounding the bone. A statistically significant enhancement was detected in the treated mice, compared to the nontreated animal, by calculating the photon count after injection and the circulation time of about 30 min, indicating the feasibility of tissue imaging and sufficient signal sensitivity of these CDs nanoprobes as effective bone-seeking agent for the prediction of bone failure, considering the crack fracture mechanics (Figure 3(b)) [119].

Various metal ions doped into pDA during the hydrothermal treatment lead to the formation of FL CDs with Em wavelengths of up to 700 nm. The Ni-pDA-CDs were prepared using pDA and nickel ions (Ni^2+^) as raw materials that exhibited Ex-independent Em (at ∼605 nm) with good photostability. A549 live cells treated with Ni-pDA-CDs for 30 min emitted strong red fluorescence under laser Ex at 552 nm in nucleoli, indicating the nucleolus targeting mechanism of Ni-pDA-CDs. Further, the *in vivo* imaging performance of Ni-pDA-CDs in tumor-bearing mice and zebrafish was investigated. The tumor region emitted bright red fluorescence after the intratumoral injection of Ni-pDA-CDs with a high signal-to-noise ratio of the tumor fluorescence. These Ni-pDA-CDs mainly accumulated in the tumor, with negligible distribution in other organs (heart, liver, spleen, lung, and kidneys), suggesting their good biosafety. Additionally, the Ni-pDA-CDs-incubated zebrafish for 30 min were well stained with bright red fluorescence, confirming that they could pass through the mucus layer and interact with the cells in zebrafish due to their ultrasmall size, positively charged surfaces, and amphiphilicity. These experiments suggest the potential of these Ni-pDA-CDs as excellent red-emissive FL nanoprobes for *in vivo* imaging in both mice and zebrafish models (Figure 3(c)) [108].

The above studies show that these FL CDs hold great promise in the bioimaging of animal models that can support efficient diagnosis and treatment in medicinal applications. Nevertheless, it is worth developing the FL CDs that exhibit excellent biocompatibility and efficient ability of clearance, providing excellent FL probes for tracking tumors, delivering drugs, monitoring the ongoing disease, and further biomedical applications. Surface modification of CDs is needed to study for the elimination of nonspecific absorption onto CDs, and specific imaging of targets *in vivo* should be considered carefully when developing CDs.

## 4. Fluorescent Carbon Dots for Bioimaging-Supported Sensing Applications

Table 2 summarizes various CD-based imaging-supported sensing applications towards different targets such as metal ions, biomolecules, pH, temperature, and polarity. Case studies of their sensing performance are then described in this section based on their target.

### 4.1. Fluorescent Carbon Dots for the Bioimaging-Supported Sensing of Metal Ions

It is worth noting that effective probes with excellent biocompatibility and photostability that can sensitively detect metal ions in living cells and *in vivo* remain a highly essential and challenging goal. Diverse CDs have been developed for the sensing applications of various ions, such as Fe^3+^, Ag^+^, Cu^2+^, and Hg^2+^. Fluorine (F)-doped CDs were successfully synthesized by a solvothermal process using difluoro-1,2-benzenediamine as the F source, and tartaric acid to improve aqueous solubility, for the intracellular detection of Ag^+^ ions. The FCDs emitted Ex-dependent Em with yellow fluorescence (maximum Ex/Em at 360–500)/550 nm and red fluorescence (maximum Ex/Em at 600/540–580 nm). F-doped CDs possessed remarkable water solubility, high biocompatibility, and excellent photostability, and could act as nanoprobes for the selective detection of Ag^+^ in HEK 293 normal cell and B16F10 cancer cell, which was confirmed by the quenching FL image in the presence of Ag^+^ (Figure 4(a)) [162].

An on/off/on FL CD-based nanosensor was successfully fabricated for in vitro and in/ex vivo Fe^3+^ detection. CDs prepared by a solvothermal treatment of glycerol and a silane molecule (N-[3-(trimethoxysilyl)propyl]ethylenediamine (DAMO) exhibited favorable biocompatibility and excellent fluorescence properties that included high QY blue fluorescence 45% at optimal Ex/Em of 350/442 nm, robust photostability in a wide range of ionic strengths and pH, selectively monitoring Fe^3+^ in Hela cells for 30 min and zebrafish for 2 h in the range 0–100 *μ*M. Herein, FL imaging of Hela cells and zebrafish after treatment with Fe^3+^ was obtained and FL intensity measured, showing the gradual decrease of intensity with increasing concentration of exogenous Fe^3+^. These CDs could semiquantitatively detect Fe^3+^*in vitro* and *in vivo*. The feasibility of these CDs for the detection of Fe^3+^*in vivo* was further evaluated through the tumor-specific imaging of nude mice bearing subcutaneous U14 xenograft tumors. Normal and tumor regions of a mouse model were imaged under *in vivo* animal imaging systems after 1 h postinjection of CDs/Fe^3+^ dots. The fluorescence intensity of the tumor region was stronger than that of normal tissue, which was verified by *ex vivo* tissue imaging, suggesting their possibility of realizing tumor-site imaging (Figure 4(b)) [126].

Amphiphilic FL carbon dots (A-CDs) were synthesized by cetyltrimethyl ammonium bromide (CTAB) modification of CDs that were prepared from CA and methionine. The fluorescence of these A-CDs was quenched by morin through electrostatic interaction between abundant amino groups of A-CDs and phenolic hydroxyl groups of morin, and then recovered in the presence of Al3+ by the release of A-CDs due to the strong complex of Al^3+^ and morin. These phenomena were used to detect Al3+ ions in HUVEC cells via cell imaging, showing fluorescence color that changed from light to deep green with increasing concentrations of Al^3+^ ions from 5–20 *μ*M [149]. Green synthesis from *Dunaliella Salina* was used to obtain strong blue FL CDs with a maximum Ex/Em at 340/415 nm at a QY of 8% for the utilization of CDs as an FL turn-off sensor for Hg^2+^ and Cr^6+^ ions in living cells. These CDs exhibited good biocompatibility, high photostability, and negligible photobleaching, making them suitable for *in vitro* cell imaging. Upon treatment of exogenous Hg^2+^ and Cr^6+^ at 100 *μ*M, the fluorescence of HEK-293 cells was strongly quenched in the red and green channels, indicating their possibility of detecting endogenous Hg^2+^ and Cr^6+^ contaminated live cells [150].

These results indicate that CDs-based bioimaging-supported sensing platforms for metal ions have been successfully developed *in vitro* and *in vivo*. However, it is required to carefully study the specificity of these CDs in sensing ions using FL imaging. Autofluorescence is considered the major issue for bioimaging of cells and tissue. Therefore, it is necessary to develop FL CDs that will not be affected by the cell and tissue autofluorescence, leading to a better possibility to recognize the targets. These reported studies are qualitative analysis for metal ions through bioimaging, which is unable to explore the minimum detectable level of ions. Therefore, quantitative analysis is required to predict the possibility of prepared CDs for practical application.

### 4.2. Fluorescent Carbon Dots for the Bioimaging-Supported Sensing of Biomolecules

Detection of the presence of small biomolecules that may be toxic or play a role in physiological processes is critical for various biomedical purposes. Amine-rich CDs with blue fluorescence were synthesized from CA and PEI and were then covalently assembled with nucleolin-targeting recognition nucleic acid aptamer AS1411 and a CTSB-cleavable peptide substrate that tethered with near-infrared (NIR) fluorophore chlorin e6 (Ce6-Pep), forming the nanoprobe AS1411–Ce6–CDs for cancer targeting and the imaging of cathepsin B (CTSB, a biomarker for malignant tumors), in living cancer cells (Figure 4(c)). Blue fluorescence of CDs at 450 nm was strongly quenched upon the conjugation with Ce6 via efficient fluorescence resonance energy transfer (FRET); otherwise, NIR fluorescence enhancement of Ce6 at ∼650 nm was observed. After being internalized into cancer cells via nucleolin-mediated endocytosis, the overexpressed CTSB in the lysosome could cleave Ce6–Pep from AS1411–Ce6–CDs to terminate the FRET process, recovering the efficient ratiometric fluorescence response toward endogenous CTSB from NIR to blue Em. Compared to no fluorescence in nucleolin-deficient HEK293 cells, significant fluorescence was observed in nucleolin-positive Hela cancer cells, confirming that AS1411 aptamer could bind to nucleolin-positive cancer cells with high specificity. Thus, these CD-based nanoprobes could be particularly suitable for monitoring the low abundance of CTBS biomarkers via precise cell imaging (Figure 4(d)) [137].

Superoxide anion (O_2_^−^) is considered one of the primary reactive oxygen species (ROS) associated with major diseases. Se- and Te-containing CDs for the detection of O_2_^−^ were successfully fabricated by the hydrothermal treatment of FO-PTe and FO-PSe as carbon sources, and their selectivity and sensitivity toward O_2_^−^ was evaluated. These Se- and Te-containing CDs exhibited the optimal Ex/Em at 440/550 nm and 380/440 nm, respectively, showing enhanced fluorescence after the reaction with O_2_^−^, and quenching when reacting with glutathione, making it possible to monitor the reversible and dynamic response of O_2_˙^−^. The feasibility of these CDs for the analysis of O_2_^−^ was investigated using two-photon fluorescence imagery of different cells (hepatocytes, HepG2 cells, macrophages, Hela cells, and lung cancer cells) and a mouse-bearing tumor model. Under 800 nm Ex, two-photon fluorescence Em of 400–500 nm for Te-CDs and 500–600 nm for Se-CDs were observed to be clearer in tumor cells than in normal cells, due to the high concentration of O_2_^−^ in cancer cells, compared to in normal cells. Additionally, brighter fluorescence with deep tissue penetration and reduced background fluorescence was obtained in the breast tumor tissue of mice compared to normal abdomen tissue due to the significantly higher level of O_2_^−^ in tumor tissue. Te-containing CDs exhibited the highest sensitivity toward O_2_^−^, suggesting that they could serve as nanoprobes for the real-time and dynamic imaging of O_2_^−^ fluxes (Figure 4(f)) [143].

Gold-carbon quantum dots (GCDs) synthesized by the modification of CDs and gold nanoclusters through a microwave-assisted method immobilized the tumor-specific antibodies to serve as FL nanoprobes for the intracellular imaging of cancer-derived exosomes. HER2, a common surface marker found on SKBR3 exosomes, was used as a target protein for the detection of exosomes in Hela cells. After being taken up by cells, the anti-HER antibody conjugated nanoprobes stuck to SKBR3 exosomes and showed bright green fluorescence in the cytoplasm, indicating the excellent intracellular fluorescence image of exosomes [147].

Coenzyme A, an important coenzyme in many biochemical reactions of the human body, such as neurodegeneration, protein acetylation, autophagy, and signal transduction, might cause different types of damage due to the deficiency of CoA. Green synthesis was conducted under hydrothermal heating using two natural biomasses (water chestnut and onion) as precursors to obtain the S and N co-doped FL CDs (S, N/CDs) that were used to monitor the presence of coenzyme A in human bladder cancer T24 cells. These S, N/CDs possessed strong blue fluorescence with maximum Ex/Em at 370/475 nm that was dramatically quenched when bound to Cu^2+^ ions and then restored fluorescence in the presence of coenzyme A due to the stronger complex between thiol groups of coenzyme A and Cu^2+^. After the loading of S, N/CDs into T24 cells for 30 min, the stronger blue and green fluorescence was observed in the T24 cells excited at 405 and 488 nm in the presence of coenzyme A, indicating that S, N/CDs-Cu^2+^ probe penetrated cell membranes, and efficiently imaged intracellular Coenzyme A [141].

Fluorescence imaging with effective monitoring of cytochrome c as an important biomarker for the early stage of apoptosis in cell apoptosis was developed using N-doped CDs that were prepared by the hydrothermal treatment of aconitic acid and tryptophan. These CDs showed strong blue fluorescence with an intensity maximum at 455 nm under 370 nm Ex and QY at 20%, which is obviously quenched by cytochrome c, facilitating the *in-situ* detection of cytochrome c for apoptosis signaling. After treatment of HepG-2 cells with N-doped CDs for 2 h, the bright blue Em was gradually decreased with increasing concentrations of etoposide, which is an apoptosis inducer to specifically trigger the release of cytosolic cytochrome c from mitochondria, indicating the quantitative imaging of etoposide-induced intracellular release during cell apoptosis. The ability to detect cytochrome c was further investigated in zebrafish imaging where brighter blue fluorescence in the abdomen of 3-day old CDs-treated zebrafish was observed, as compared to that when the zebrafish were consequently treated with cytochrome c, suggesting N-doped CDs as effective FL nanoprobes for the monitoring of cytochrome c mediated cell apoptosis pathway (Figure 4(e)) [142].

Overall, there are several excellent CDs that have been used to detect biomolecules *in vitro* and *in vivo* via bioimaging. Again, autofluorescence of cells and tissue, and the specificity of FL CDs must be carefully considered to enhance the sensing performance. Quantitative analysis should be studied for further practical application. The cytotoxicity of CDs is an urgent matter to investigate before the sensing process. The time and mechanism of CD penetration into the target should be clearly examined for further effective imaging-supported sensing application.

### 4.3. Fluorescent Carbon Dots for the Bioimaging-Supported Sensing of pH, Temperature, and Polarity

The direct measurement of some intracellular conditions in cells is essential but not easily achieved, making it difficult to explain their effects on bioreactions. The dual-Em CDs obtained by the hydrothermal pyrolysis of aniline blue (AB) and rhodamine B (RhB), and CDs made from CA and 1,4-butanediamine in the presence of PEG 400, denoted as RhB-AB-CDs, were exploited as intracellular pH nanoprobes in the mycelia of Pholiota adipose fungus. These RhB-AB-CDs emitted two distinct Em bands at the maximum Ex/Em of 380/443 nm and 400/580 nm, which were attributed to the Ex-dependent Em of CDs and the Ex-independent Em characteristic of RhB, respectively, making the signal sensitive to pH, corresponding to the ratio of Em intensity at 580 and 467 nm under Ex at 400 nm. They were then applied to monitor the intracellular pH of fungal mycelia using the ratio of FL intensity in the red/blue channels at 580/467 nm under continuous Ex at 405 nm, showing the increase of this ratio with an increase of pH value from pH = 5.52 to 7.50 with good linear regression of 0.997, suggesting the highly photostable fluorescence of these CDs for the reliable long-term monitoring of intracellular pH (Figure 5(a)) [172].

Temperature is also an important factor in the life process, due to the role of thermal energy transfer in all biological reactions in organisms. Faint yellow fluorescence CDs were synthesized directly from ascorbic acid aqueous solution by an electrochemical method at RT and exhibited Ex-dependent Em with a maximum Ex at 400 nm. The fluorescence of these CDs with a high quantum yield at 35.2% was stable with different pH values, ionic strengths, and storage times, and sensitive to temperature, with the fluorescence intensity changing linearly with a temperature of 20–100 °C. Human normal HEK 293T cells emitted faint yellow fluorescence under 405 nm irradiation; moreover, as the temperature increased from 20 to 40 °C or decreased from 40 to 20°C, the fluorescence intensity gradually decreased or increased, respectively. Furthermore, these CDs can especially stain the nucleolus by entering the cell nucleolus and adsorbing on nucleic acids (DNA and RNA). Thus, the CDs could act as an effective nanothermometer to monitor in vitro and in vivo temperature by utilizing the yellow-emissive nanoprobes of nucleolus specific imaging (Figure 5(b)) [174].

Monitoring the change of intracellular polarity plays a great role in the understanding of its functions in live cells, due to its large impact on the activity of biomolecules or the function of domains. The FL carbon dots R-CDs with a 5 nm spherical shape and good monodispersity were successfully obtained through a hydrothermal method at 200°C for 12 h using p-phenylenediamine as a precursor, displaying significant red Em under 420 nm Ex, and were then utilized as FL nanoprobes for the real-time sensing of polarity in living cells. The R-CDs possessed a high quantum yield of 47.87%, high photostability, good biocompatibility up to 400 *μ*g/mL, and dual targetability for mitochondria and lysosomes in cells. Various solutions with increasing polarity from 10 to 99 % were obtained by mixing water and dioxane based on volume ratios and showed a decrease in FL intensity of up to 11-fold. For colocalization examination of these R-CDs, human liver cancer HepG2 cells costained with R-CDs, Mito-tracker green, and Lyso-Tracker Red presented partial overlaps of the regions between the red FL of R-CDs and the Mito-tracker green or Lyso-Tracker Red areas, suggesting the preferential accumulation of R-CDs in mitochondria and lysosomes. The ability of R-CDs to monitor the polarity change in HepG2 cells by the reduction of red-emissive fluorescence with increasing polarity was successfully studied. Interestingly, the imaging of HepG2 cells and normal human liver HL-7702 cells both treated with R-CDs showed the difference between the strong red fluorescence in HepG2 cells and weak fluorescence in HL-7702 cells, discriminating the lower polarity in cancer cells with high polarity in normal cells. These R-CDs nanoprobes could contribute to mitochondrial and lysosomal polarity-related studies (Figure 5(c)) [173].

## 5. Fluorescent Carbon Dots for Bioimaging-Guided Therapeutic Application

Table 3 summarizes the imaging-guided therapeutic approaches using various CDs, including individual treatment (chemotherapy, photodynamic therapy, photothermal therapy) and combined treatment. Case studies of this CD-based imaging-guided therapy are then deliberated in this section based on their biotargets and performance.

As fluorescence nanoprobes, CDs have been widely investigated to enhance fluorescence imaging-guided therapeutics for the better intervention of tumors. Using folic acid (FA) that shows high receptors in hepatoma cells and DOX as an anticancer drug, FA-CDs-DOX with a high fluorescence quantum yield (97%) was synthesized to enhance the antitumor activity and imaging efficiency for imaging-guided chemotherapy of targeted liver cancer. *In vivo* images of tumor-bearing mice after the injection of FA-CDs-DOX displayed strong orange-red fluorescence under Ex at 480 nm light, while no FL signal was observed in tumor-bearing mice treated with CDs or DOX only, indicating their ability to penetrate tumor tissue and skin to achieve FL imaging effects. This FA-CDs-DOX also exhibited significantly higher tumor inhibition *in vivo* through the targeting ability of FA-CDs-DOX compared to that of free DOX, suggesting the effective improvement of FL image-guided chemotherapeutic effect in liver cancer therapy (Figure 6(a)) [182].

Innovative nanomedicine for the theranostics of multidrug-resistant (MDR) tumors remains a challenge for scientists. Yellow FL CDs (y-CDs)/dendrimer nanohybrids have been developed as a platform for ultrasound-enhanced fluorescence imaging and chemotherapy of MDR tumors (Figure 6(b)). These nanoprobes were prepared via electrostatic interaction between y-CDs and generation 5 (G5) poly(amidoamine) dendrimers and d-*α*-tocopheryl polyethylene glycol 1000 succinate (G5-TPGS), then physically loaded with anticancer drug doxorubicin (DOX) to form (G5-TPGS@y-CDs)-DOX complexes with high drug loading efficiency of 40.7%. The tumor fluorescence imaging by these complexes with a strong Em peak at 550 nm was further evaluated in the presence and absence of ultrasound-targeted microbubble destruction (UTMD). Images of i*n vivo* mice-bearing MCF-7/ADR xenografts after the intravenous injection of y-CDs and (G5-TPGS@y-CDs)-DOX complexes (with or without UTMD) displayed stronger fluorescence signals in the tumor region, even at 6 h postinjection, compared to weaker fluorescence in the y-CDs control group, due to the quick metabolization of small free y-CDs. Significant enhancement of fluorescence was observed stably in the tumor region with the assistance of UTMD *in vivo*, as well as *ex vivo*, tumor and other organs, supporting the enhancing role of the UTMD-rendered sonoporation effect. There was no obvious inhibition effect on the tumor growth of UTMD, thus bioimaging-guided treatment with (G5-TPGS@y-CDs)-DOX with the support of UTMD was further investigated, demonstrating the effective therapeutic effect of this CD-based platform for MDR tumor chemotherapy (Figure 6(c)) [178].

On the other hand, multicolor highly crystalline carbon nanodots (HCCDs) were successfully fabricated for the use in dual-modal imaging-guided PTT of glioma. HCCDs exhibited optimal Ex/Em 440/506 nm with Ex-dependent full-color fluorescence, where the Em was tuned from blue to green through increasing the Ex wavelength. With high water dispersity and good biocompatibility, U87 glioma-bearing mice were treated with HCCDs for the investigation of imaging-guide PTT performance, displaying that intravenously administrated HCCDs gradually accumulated in the tumor, emitted the brightest imaging at 30 min postinjection under 465 nm Ex, and achieved the effective PTT effect under an 808 nm laser. The capacity of HCCDs to permeate the glioma and specifically accumulate in glioma cells could provide imaging-guided PTT targeted to glioma in mice, without side effects to the normal tissues (Figure 6(d)) [189].

The therapeutic approach of combination phototherapy, including photodynamic therapy (PDT) and photothermal therapy (PTT), has recently shown great promise for efficient cancer therapy by inducing reactive oxygen species (ROS) or heat into tumors to kill cancer cells. The yellow FL CDs with optimal Ex/Em 500/570 nm were easily obtained by the hydrothermal treatment of 1,3,6-trinitropyrene and possessed a strong ability to simultaneously generate singlet oxygen (^1^O_2_) (QY 5.7%), hydroxyl radical (OH.), and heat effect under a 635 nm laser irradiation (73.5% photothermal conversion efficiency). Interestingly, these CDs exhibited one-photon excited (OPE) and two-photon excited (TPE) fluorescence at a peak of 570 nm and displayed green fluorescence imaging in Hela cells under excitation by both 457 and 800 nm lasers, confirming the selective accumulation of CDs in lysosomes by the overlapping fluorescence of commercial lysosome targeting dye. With good biocompatibility, *in vivo* photoacoustic imaging and the photothermal performances of CDs on the 4T1-tumor-bearing nude mice were studied after the intravenous injection of CDs for 4 h, showing significant enhancement of the PA signal in the tumor region and an increase in temperature up to 70°C under an 800 nm laser, suggesting that these CDs could act as lysosome-targeting phototheranostic agents for simultaneous PA and fluorescence imaging-guided PDT/PTT [181].

The magneto-fluorescent CDs prepared by the hydrothermal treatment of a mixture of poly lysine, CA, and GdCl_3_ were decorated on carbon nanotubes (CNTs)/doxorubicin (DOX) nanocomposites, then conjugated with FA to form FA-GdN@CDs-CNTs to serve as dual-modal fluorescence/magnetic resonance (MR) imaging. These CD-based complexes possess low toxicity, good biocompatibility, and drug release ability forced by pH and NIR light and are suitable for synergistic chemo-photothermal therapy (Chemo/PTT) in cancer excision. Fluorescence images of HeLa cells treated with FA-GdN@CDs-CNTs displayed green and red fluorescence under 488 and 543 nm illumination in cell membrane and cytoplasm, but not in nuclei, indicating that this complex could internalize in cell membranes, and enter HeLa cells via endocytosis. With the support of FL imaging, the combined chemo-PTT in HeLa tumor-bearing nude mice was effective in reducing the tumor with a great contribution to tumor inhibition, without damage to major organs [191]. Overall, owing to the high tumor-inhibition efficacy and low side effects, the capability of the CD imaging-guided therapeutic was proven as a smart approach for enhanced therapeutic effects, suggesting it offered an excellent strategy for potential clinical therapeutic application.

This section indicates that CDs exhibit the promising potential for FL imaging-guided therapy due to their unique properties. Compared to other CDs, the red-emissive CDs possess a more efficient capability to serve as theragnostic nanoagents *in vivo*. Surface modification of CDs is essential to precisely consider for reducing the non-specific protein absorption and improving the specifically tumor-targeted ability. The cytotoxicity and perfect ability of clearance must be attentively investigated for the best therapeutic efficacy without any side effects. It is becoming necessary to develop CDs with both high FL quantum yield and synergistic chemo/PDT/PTT, suggesting that CDs could be a promising theragnostic candidate for imaging-guided therapy.

## 6. Conclusions and Perspectives

Recently, fluorescent carbon dots have greatly accelerated the advancement of bioimaging-supported nanomedicine to supply efficient biomedical applications, including the efficacy of molecular imaging that increased the image properties over the conventional FL agents, accurate monitoring of the presence of ions and molecules via imaging for biological and medical studies, and efficient treatment of tumors via FL imaging guidance. As discussed above, various reports have successfully developed multicolor FL CDs with superior properties, such as high fluorescence, excellent photostability, ease of functionalization, and good biocompatibility, that have been utilized in multiple biomedical applications, from biology to medicine. Although the advancement of CD-supported imaging-based nanomedicine holds promising potential in further clinical medicine, some critical aspects require more attention before shifting to the clinical setting.

Even though the affordability of CDs was confirmed, their exploitation in imaging-supported nanomedicine is difficult to offer globally, due to the limitation that the large-scale synthesis methods of functional CDs have not been standardized. Because fluorescence is the main property of CDs for imaging-supported medicine, the high quantum yield of CDs must be obtained for the best performance of bioimaging. For example, the high quantum yield of CDs can be achieved by heteroatom doping [198]. Although research on the toxicity of CDs has confirmed their biocompatibility *in vitro* and *in vivo*, the long-term accumulation of CDs in targeted tissue or organs might cause irritation, inflammation, renal toxicity, hepatotoxicity, and immune system problems in organisms. They remain challenges for scientists to evaluate the possibility of CDs *in vivo*, and the release capacity of CDs out of the body, without side effects. Sufficient photostability of CDs must be ensured to analyze the stability of the FL signal for further *in vivo* applications.

In the field of bioimaging-supported sensing platforms for abnormal metal ions and molecules, almost all reports could only obtain qualitative detection or semiquantitative monitoring in the microgram range; hence, accurate quantitative detection should be acquired to provide significant information about biological processes or the diagnosis and prognosis of diseases. Specific organelle-targetable CDs possess the ability to image the selective targets, distinguish cancerous cells from normal cells, or detect further biomarkers in the targeted organelles. Thus, the selection of optimal CDs for specific imaging-supported applications is highly required for the improvement of sensing performance. Further, the high specificity of the bioimaging-supported sensing platforms should also be improved in the presence of various interferences in the organism's body.

For FL imaging-guided therapy, the assurance of tumor-targeted specificity that will be increased through image resolution and performance is required for the tracking of tumors during the therapeutic process. This tumor specificity is attributed to the loading optimization of specific agents towards each tumor target, the stability of conjugated nanoprobes in the body, and the improvement of FL microscopic techniques through the enhancement of contrast-to-noise ratio. Overcoming the nonspecific uptake in nontargeted organs for the best treatment of tumors should be concentrated on. CDs that can generate FL signals from deeply located tissue should continue to be developed to enhance the visualization capacity of CDs in deep tumor tissue. In addition, the CDs with highly biodegradable ability must be considerably focused on to develop facile utilization in clinical medicine without side effects. Based on the ease of functionalization of CDs, combined therapeutic approaches, such as chemo/PDT/PTT, which can achieve more efficacious treatment, should be integrated. For fighting bacterial infections, CDs-integrated biofilms were successfully utilized for imaging and selectively eliminating bacteria, suggesting that the integration of CDs along with antibiotics in biofilms could exhibit better control of bacterial infections than alone [199]. Hence, CDs-integrated materials should be intensively developed for their efficacy enhancement. Furthermore, technical professionals for accurate biomedicine are also important, so that medical scientists will have sufficient medicinal skills to perform the techniques and analyze the acquired data for thorough implementation.

In summary, the applications of CDs in FL imaging-based biomedicine appear to hold promising innovation for further clinical use. Although these CD-supported imaging-based biomedicines have been reported in the initial stages, their substantial potential will be achieved in clinical medicine if their possibility is successfully evaluated in clinical trials. The toxicology, pharmacokinetic, and applicable studies of these CD-based imaging-supported biomedicine concepts in the human body should be intensively researched. The development of advanced CDs for these emerging biomedicine concepts is being completed day-by-day, leading to the realization of real medical accomplishment in the near future. Due to the superior properties of CDs in the fields of imaging-based biomedicine, their enormous applications could be proficiently handled globally for the best medicinal intervention.

## Figures and Tables

**Figure 1:** Diverse imaging-supported biomedical applications using fluorescent carbon dots include the FL imaging of various biotargets (different targeted cells, tissues, fungi, bacteria, and animals), FL imaging-supported sensors (metal ions, biomolecules, pH, thermal, polarity), and FL imaging-guided therapy (chemotherapy, photothermal therapy, photodynamic therapy, and combined therapy).

**Figure 2:** *In vitro* FL imaging of various targets using CDs. (a) CLSM images of CDs-treated SiHa cells. (A) Bright-field image, (B)–(E) multicolor FL images from blue, green, yellow, and red under excitation/emission wavelengths of ((405/422 ± 25), (488/500 ± 25), (515/570 ± 25), and (543/650 ± 25)) nm, respectively, adapted with permission from Ref. [25]. (b) Washfree selective nucleus imaging of Hela cells through hydrogen-bonding-induced emission, adapted with permission from Ref. [61]. (c) Selective lysosomal imaging of live Hela cells confirmed by well-overlapped image of CDs (collected at (420–580) nm) and Lyso-Tracker Red (commercial lysosomal probe, collected at (650–800) nm) in Hela cells under 405 nm excitation, adapted with permission from Ref. [70]. (d) Mitochondrial imaging of MCF-7 cells incubated with CDs (Ex: 488 nm), and then MitoTracker (Ex: 638 nm), ER-Tracker (Ex: 552 nm), Golgi-Tracker (Ex: 552 nm), or LysoTracker (Ex: 552 nm), confirmed by the coincident overlay between CDs green FL and MitoTracker red FL, but not ER-Tracker, Golgi-Tracker, or LysoTracker, adapted with permission from Ref. [63]. (e) Red-emissive FL imaging of different plant tissues through the selective cellulose-binding of CDs, adapted with permission from Ref. [81]. (f) CLSM images of the CDs FL monitoring of *S*. *aureus* and *E*. *coli* at various incubation periods, adapted with permission from Ref. [15]. (g) Differentiation of gram-positive *S*. *aureus* bacteria from gram-negative *E*. *coli* bacteria using CLSM images of a mixture of CDs-treated bacteria under 405 nm excitation, adapted with permission from Ref. [14]. (h) CLSM images of *C. gloeosporioides* fungus labeled by different color CDs, adapted with permission from Ref. [99].

**Figure 3:** *In/Ex vivo* FL imaging of animals using CDs. (a) Real-time *in vivo* red FL images in nude mice at different time periods after (A) subcutaneous, and (B) intravenous injections of CDs via the tail vein revealed the accumulation of CDs in the tumor tissue. Adapted with permission from Ref. [107]. (b) *In vivo* FL of monophosphonated CDs in the tibia of (A) non-treated mice, (B) treated mice (Ex/Em = 430/600 nm); (C) treated the animal with the computed tomography-fused fluorescence image (Ex/Em = 465/700 nm), showing the feasibility of CDs for the detection of bone microcracks. (D) Significant difference of FL radiance between CDs-nontreated and CDs-treated mice (^*∗*^*p* value < 0.05). Adapted with permission from Ref. [119]. (c) (A) *In vivo* FL images, and (B) corresponding FL intensity of the tumors before and after the intratumoral injection of CDs for different time periods. (C) *Ex vivo* FL images, and (D) corresponding FL intensity of different organs of mice after CDs injection for different day periods (^*∗∗*^*p* value < 0.01, ^*∗∗∗*^*p* value < 0.001). (D) CLSM image, and (E) bright-field image of CDs-stained zebrafish. Adapted with permission from Ref. [108].

**Figure 4:** Fluorescence imaging-supported sensing of various metal ions and biomolecules. (a) Intracellular silver ions detection in HEK 293T cells and B16F10 cells without (-), and with (+) Ag^+^, through obvious quenching phenomenon. Adapted with permission from Ref. [162]. (b) *In vivo* semiquantitative detection of Fe^3+^ through CLSM images of zebrafish treated with CDs and quenching FL effect after treatment with different concentrations of Fe^3+^ and corresponding FL intensity. Adapted with permission from Ref. [126]. (c) Action mechanism of AS1411–CQDs–Ce6 nanoprobe for the intracellular detection of endogenous CTSB through specific binding of AS1411 aptamer with nucleolins. Adapted with permission from Ref. [137]. (d) Strong FL imaging of living HeLa cells under different treatments with AS1411–CQDs–Ce6 and no FL signal of nucleolin-deficient HEK293 cells under treatment with AS1411–CQDs–Ce6 indicated the feasibility of nanoprobes for the detection of CTSB. Adapted with permission from Ref. [137]. (e) *In vivo* detection of Cyt (c) in zebrafish. CLSM images of zebrafish (A) untreated NCDs, (B) incubated with NCDs for 30 min; and subsequent treatment with (C) Cyt (c), or (D) etoposide for 20 min showed a significant FL quenching effect of Cyt (c). Adapted with permission from Ref. [142]. (f) Selective detection of superoxide anion in mice through the FL enhancement of O_2_−to CDs. FL imaging of O_2_−levels in the tumor tissues (A)–(C) and normal tissue (D)–(F) after treatment with Te-CDs, FO-PTe, and Se-CDs-treated mice, respectively, acquired using 800 nm two-photon excitation. (G) Corresponding FL intensity revealed the significant increase of O_2_−level between normal and tumor tissues. Adapted with permission from Ref. [143].

**Figure 5:** Fluorescence imaging-supported sensing of other effects (pH, thermal, polarity). (a) Response mechanism to pH of RhB-AB-CDs based on the inner filter effect of Aniline Blue on the emission of Rhodamine B and fluorescence color changes of CLSM images of RhB-AB-CDs-treated Pholiota adipose mycelia at pH of (5.5 to 7.5). Adapted with permission from Ref. [172]. (b) (A) Fluorescence linear relationship CDs during heating and cooling processes. (B) Thermal stability of FL lifetimes over seven cycles of heating and cooling between (30 and 70) °C ((I)_0_ and (I) are the FL intensity at 20°C and other temperatures, respectively). (C) CLSM images of CDs-treated 293T cells at (20, 30, and 40)°C; Em was collected at (415–550) nm at an excitation wavelength of 405 nm. Adapted with permission from Ref. [174]. (c) Intracellular polarity sensor through FL images of HepG2 cells incubated with (A) DMSO + CDs (obvious FL enhancement), (B) CDs, and (C) HBSS + CDs (quenching FL) at Ex/Em of 488/(550–650) nm. Adapted with permission from Ref. [173].

**Figure 6:** Fluorescence imaging-guided therapy using CDs. (a) Schematic of FL imaging-guided therapeutics of liver cancer using FA-CDs-DOX. Adapted with permission from Ref. [182]. (b) Demonstration of ultrasound-enhanced theranostics of multidrug-resistant tumors using G5-TPGS@y-CDs)-DOX drug-loaded CD/dendrimer nanohybrids. Adapted with permission from Ref. [178]. (c) (A) Therapeutic schedule of (G5-TPGS@y-CDs)-DOX and ultrasound-targeted microbubble destruction (UTMD) treatment *in vivo*. (B) Tumor volumes, (C) body weights, and (D) survival rate of mice after intravenous injection periods of different groups (saline, free DOX, (G5-(m)PEG@y-CDs)-DOX, (G5-TPGS@y-CDs)-DOX, or (G5-TPGS@y-CDs)-DOX + UTMD) showed the effective chemotherapy of tumors. Adapted with permission from Ref. [178]. (d) *In vivo* FL images of glioma-bearing mice after intravenous injection of saline and HCCDs, and *ex vivo* images of major organs after administration under 465 nm excitation displayed the accumulation of HCCDs in the tumor region for the effective FL imaging-guided PPT of glioma. Adapted with permission from Ref. [189].

**Table 1:** *In vitro* and *in vivo* bioimaging applications using FL CDs.

Precursors/Forms	FL Color	Applied Ex/Em (nm)	Microscopic	Application	Biotarget	Ref.
Ethylenediamine (EDA) into yeast extract solution	Green	405/–	CLSM	Bacterial viability evaluation	*E. coli, S. aureus*	[13]
Si-QAC, glycerol	Blue	360/473	CLSM	Gram-type identification	*S. aureus, M. luteus, B. subtilis*	[14]
				Gram-positive antibacterial		
Pluronic F-127, 4-chlorophenylboronic acid	Blue	380/400	CLSM	Detection of glucose-containing bacteria	*E. coli, S. aureus*	[15]
Tulsi leaves	Blue/Yellow/Red	360/435	FM	Imaging of bacteria	*E. coli, B. subtilis*	[16]
Choline bicarbonate, oleic acid	Blue–red	300–500/416–556	FM	Imaging of bacteria	E. coli, Vibrio owensii, Bacillus cereus, and Vibrio alginolyticus	[17]
Roasted grams	Blue–red	320–500/475–610	FM	Imaging of bacteria	*E. coli*	[18]
Beer yeast	Blue	405/–	CLSM	Bacterial viability evaluation	*E. coli*	[19]
	Green	488/–		Imaging of dead bacteria		
	Red	555/–				
Thiourea, TAE	Blue	380/430–470	FM	Imaging of bacteria, cells	E. coli, Pseudomonas, Staphylococcus, Klebsiella, and hBEC	[20]
	Green	450/510–560				
	Red	505/585–640				
3-Aminophenylboronic acid, CA	Blue	360/420	CLSM	Imaging of cells	Hela	[21]
Collagen	Blue	370/–	Two-photon CLSM	Imaging of cells	RL-14	[22]
	Green	490/–				
	Red	550/–				
CA, urea, cupric chloride	Blue	405/–	CLSM	Imaging of cells	MCF-7	[23]
	Green	488/–				
	Red	543/–				
CA, PEI	Blue	405/–	CLSM	Imaging of cells	3T3	[24]
	Green	488/–				
EDA, H_3_PO_4_	Blue	405/422	CLSM	Imaging of cells	SiHa	[25]
	Green	488/500				
	Yellow	515/570				
	Red	543/650				
Aconitic acid, EDA	Blue	360/450	FM	Imaging of folate receptor-overexpressed cells	Hela, SMMC-7721	[26]
Sucrose, EDA, and H_3_PO_4_	Blue	402/–	CLSM	Imaging of cells	HepG2 cells	[27]
	Green	488/–				
	Red	543/–				
ATP, LaCl_3_	Blue	350/460	CLSM	Imaging of cells, tissue	A549, nude mice	[28]
	Green	488/500				
	Red	543/650				
D-Arginine, 4-Methylumbelliferone	Blue	378/452	CLSM	Imaging of cells	MC3T3	[29]
Resorcinol, EDA	Blue	230/326	CLSM	Imaging of cells	OVCAR-3, MCF-7	[30]
	Green	230/443				
	Yellow					
	Red					
Watermelon juice, ethanol	Blue	355/439	CLSM	Imaging of cells	HepG2	[31]
Crab shells	Blue	360/450	CLSM	Imaging of cells	Hela	[32]
Diammonium hydrogen citrate, PEG-400	Blue	370/432	CLSM	Imaging of cells	BGC-823, CT26.WT	[33]
CA, dethylene glycol bis (3-aminopropyl) ether	Blue	300/440	FM	Imaging of tissue	Glioma	[34]
Lily bulbs	Blue	370/448	FM	Imaging of cells	A549	[35]
Succinic acid, glycerol	Blue	280–480/410–525	FM	Imaging of cells	KKU213	[36]
	Green					
Metformin hydrochloride, glucose anhydrous	Blue	480/–	FM	Imaging of cells	CT26.WT	[37]
	Green	560/–				
	Red	720/–				
Urea, PEG	Blue	405/–	CLSM	Imaging of cells	L929	[38]
	Green	488/–				
	Red	543/–				
Saffron	Green-blue	400/485	FM	Imaging of cells (rat)	Olfactory mucosa cells	[39]
					Bone marrow cells	
Alendronate sodium	Blue	405/–	FM	Imaging of cells	BT474	[40]
	Green	488/–				
EDA, starch	Blue	405/420–510	CLSM	Imaging of cells	BHK	[41]
	Green	405/490–560				
	Red	405/590–750				
Apple	Blue	380/490	FM	Imaging of cells	MDA-MB-231, A549, and HEK-293	[42]
Hongcaitai	Blue	405/–	CLSM	Imaging of cells	HepG2	[43]
	Green	488/–				
	Red	559/–				
CA, melamine	Blue	405/–	CLSM	Imaging of cells	HepG2	[44]
	Green	488/–				
	Red	559/–				
CA, p-phenylenediamine, borax	Blue	315/–	FM	Imaging of cells	HepG2	[45]
	Green	445/–				
	Yellow	485/–				
	Red	515/–				
						
Tartaric acid, urea	Blue	–	CLSM	Imaging of cells	MDA-MB-231	[46]
	Green					
	Red					
Acidic cotton linter waste	Blue	390/446	FM	Imaging of cells	H2452, HUVEC	[47]
	Green	482/532				
	Red	586/646				
Quince fruit	-	480/518	FM	Imaging of cells	HT-29	[48]
1,6-hexanediamine	Blue	410/–	CLSM	Imaging of cells	MCF-7	[49]
Dihydrochloride, dimethyl sulfoxide	Green	460/–				
	Yellow	480/–				
	Orange	530/–				
Citrus fruit peels	Green	330–385/–	FM	Imaging of cells	MCF-7	[50]
	Yellow	450–480/–				
	Red	510–550/–				
Gum olibanum resin	Green	420–495/525	FM	Imaging of cells	B16F10	[51]
Adenosine disodium triphosphate	Red	543/–	CLSM	Imaging of cells	HeLa	[52]
CA, EDA, arginine	Blue	330–380/–	FM	Imaging of cells	NIH 3T3, HEK 293, Hela, and MCF-7	[53]
	Green	460–495/–				
	Red	530–550/–				
Thiourea, CA, D-Glucosamine hydrochloride, and triethylamine	Green	368/505	FM	Imaging of cells	HepG2, HL-7702	[54]
Food waste	Blue	360/435	FM	Imaging of cells	HCT116	[55]
Sugarcane	Blue	405/410–460	CLSM	Imaging of cells	DU145, MCF-7, and A375	[56]
	Green	488/–500–530				
	Yellow	515/–530–570				
	Red	559/–575–675				
Hyperbranched polysiloxane	Blue	320–380/440	FM	Imaging of cells	Mouse osteoblast	[57]
Prunus cerasifera fruits	Blue	405/450	FM	Imaging of cells	HepG2	[58]
	Green	488/–				
Ginkgo fruits	Blue	405/–	CLSM	Imaging of cells	HeLa	[59]
	Green	488/–				
Triethylenetetramine, phenylenediamine	Green	360/510	CLSM	Imaging of cellular RNA	HEp-2	[60]
m-phenylenediamine, FA	Green	405/480–580	CLSM	Imaging of cell nucleolus	HeLa	[61]
CA, PEI	Blue	405/–	CLSM	Imaging of cells	HEK293	[62]
	Green	488/–				
	Red	561/–				
Chitosan, EDA, mercaptosuccinic acid, and CD-RB	Green	532/550	CLSM	Imaging of mitochondrial-targeted cells	MCF-7	[63]
Polyacrylic acid, EDA	Blue	356/520	FM	Imaging of cells	EM-6	[64]
CDs@SiO_2_	Green			Imaging of tissues	Onion bulb epidermal tissue	
PEI, 4-formylphenylboronic acid	Blue	360/462	FM	Imaging of cells	Hela	[65]
CEL powder	Blue	320/400	CLSM	Imaging of cells	Hela	[66]
	Green	400/–				
	Red	480/–				
CA,	Red	488/678	CLSM	Imaging of EGFR-overexpressed cells	HCC827	[67]
5,10,15,20-tetrakis(4-aminophenyl)porphyrin (TAPP)					MDA-MB-231	
CA, guanidine carbonate	Green	800/480	Two-photon FM	Imaging of cells	Hela	[68]
				Imaging of tissues	Rat liver tissue	
Carbon powder, ammonia	Blue	405/–	FM	Imaging of cells	HeLa	[69]
	Green	488/–				
	Red	563/–				
						
CA CDs-PEI-ML	Green	405/420–580	CLSM	Imaging of lysosome-targeted cells	Hela	[70]
Starch, L-tryptophan, and CD-MIPGlcA	Blue	371/452	CLSM	Imaging of hyaluronan-targeted cells	HaCaT, HeLa	[71]
	Green	445/500				
p-phenylenediamine, aspartic acid	Yellow	410/535	CLSM	Imaging of cells	MIDA-MB-231, MIDA-MB-68, and RPE1	[72]
Na2EDTA, GdCl3, YbCl3, and L-arginine	Blue	340/418	FM	Imaging of cells	HeLa	[73]
DL-malic acid	Cyan	405/–	CLSM	Imaging of cells	Trout gill epithelial cells.	[74]
	Purple	488/–				
	Green	514/–				
	Red	561/–				
Carbon glassy, PEG-200	Green	405/420–637	CLSM	Imaging of cells	HT29, A549	[75]
CA, EDA, GdCl3, and YbCl3	Blue	405/450	CLSM	Imaging of cells	Hela, NIH-3T3, and CHO	[76]
Adenosine triphosphate, graphene oxide	Green	488/–	CLSM	Imaging of cells	A549	[77]
	Red	543/–		Imaging of bacteria	S. aureus	
CA, PEI, GdCl3, and DTPA	Blue	354/445	FM	Imaging of cells	HeLa	[78]
CA, thiourea, and 3-amino phenyl boronic acid	Blue	405/–	CLSM	Imaging of cells	HepG2, L929	[79]
	Green	488/–				
	Red	546/–				
ZIF-8	Green	405/503	CLSM	Imaging of cells	HeLa	[80]
p-phenylenediamine	Orange	514/633	CLSM	Imaging of tissues	*Arabidopsis thaliana* leaf	[81]
PEI600, poly(tetrafluoroethylene)	Blue	348/460	CLSM	Imaging of cells	HeLa, 7702	[82]
Polythiophene phenylpropionic acid	Red	543/610	CLSM	Imaging of cells	HeLa	[83]
Cds@Au						
L-asparagine	Blue	370/449	CLSM	Imaging of cells	HeLa	[84]
CA, urea, and laurylamine	Blue	360/430	CLSM	Imaging of lysosome-targeted, endoplasmic reticulum-targeted cells	MCF-7	[85]
Bamboo leaves	Green	488/–	CLSM	Imaging of cells	HeLa	[86]
CDs-CBBA-Dox				Imaging-guided chemotherapy		
p-phenylenediamine, phosphoric acid, and Mn(OAC)_2_	Red	530/600	CLSM	Imaging of cells	B16F1, HeLa	[87]
o-phenylenediamine	Yellow, Green	465/570	FM	Imaging of cells	HepG2	[88]
CA, EDA, and ginsenoside Re	Blue	360–380/–	FM	Imaging of cells	A375	[89]
	Green	460–480/–				
	Red	510–530/–				
AEAPMS	Green	473/–	FM	Measurement of cells	Macrophages	[90]
GNR@SiO2@CD						
m-Phenylenediamine	Blue	360/444	CLSM	Imaging of cells	MCF-7	[91]
o-Phenylenediamine	Yellow	450/533				
p-Phenylenediamine	Orange	530/574				
Poly(vinylpyrrolidone), L-cysteine	Blue	350–400/420–470	CLSM	Imaging of cells	Tramp C1	[92]
	Green	460–490/520				
	Red	510–550/590				
Platanus biomass	Blue	360/476	CLSM	Imaging of cells	HeLa, L02, and macrophages	[93]
Cyanobacteria powder	Green	405/–	CLSM	Imaging of cells	PC12	[94]
Diammonium hydrogen citrate, urea	Green	420/537	CLSM	Imaging of cells	HeLa	[95]
CA, EDA	Blue	405/–	CLSM	Imaging of cells	CNE-1, HEK-293T	[96]
	Green	488/–				
	Red	640/–				
L-cystine, o-phenylenediamine	Orange	560/595	CLSM	Imaging of cells	293T	[97]
	Red	560/628				
Protamine sulfate, PEG	Blue	405/–	FM	Imaging of cells	HEK-293	[98]
	Green	488/–				
	Red	594/–				
Methyl red, EDA	Blue	–/470	CLSM	Imaging of fungi	*C. gloeosporioides*	[99]
	Green	–/511				
	Yellow	–/530				
Acacia concinna	Blue	405/–	CLSM	Imaging of fungi	*Penicillium sp.*	[100]
	Green	488/–				
	Red	561/–				
Manilkara zapota	Blue	350/443	CLSM	Imaging of bacteria	*E. coli*	[101]
	Green	420/515		Imaging of fungi	*Aspergillus aculeatus, Fomitopsis sp.*	
	Yellow	440/563				
L-cysteine, m-PD	Green	488/>515	FM	Imaging of nucleolus	MGC-803, Mel-RM, H7, HeLa, and SKOV3	[102]
				Cancer/normal cell differentiation	GES-1, FB, and HEM-d	
CA, urea	Yellow	542/612	CLSM	Imaging of nucleolus	HeLa cells	[103]
Carbon NPs, p-phenylenediamine	Green	488/500–560	CLSM	Imaging of nucleolus dsDNA	HeLa, A549	[104]
	Red	543/570–650		Imaging of nucleolus ssRNA	*C. elegans*	
				dsDNA/ssRNA differentiation		
Tris(hydroxymethyl)aminomethane, betaine hydrochloride	Red	520/600	*In vivo* imaging system	Imaging of stem cells	Human mesenchymal stromal cells - mice	[105]
*P. acidus* fruit	Blue	400/–	FM	*In vivo* imaging of nematode	*C. elegans*	[106]
	Green	470/–				
	Red	550/–				
p-phenylenediamine PDA@N-CDs(Mn)	Red	550/620	*In vivo* imaging system	*In vivo* imaging of tumor	A549 tumor-bearing mice	[107]
p-phenylenediamine, NiCl2Ni−pPCDs	Red	520/605	CLSM	Imaging of nucleolus-targeted cells	A549	[108]
			*In vivo* imaging of tumor	*In vivo* imaging of tumor	Zebrafish	
					U14 tumor-bearing mice	
Coal tar CDs-liposome	Orange	535/605	CLSM	Imaging of cells	HeLa	[109]
			*In vivo* imaging system	*In vivo* imaging of tumor	HeLa tumor-bearing mice	
Carbon nanopowder, EDA, and glycerin	Green	400/486	FM	Imaging of bone	Zebrafish	[110]
Aniline, EDA, urea	Green	410/510	FM	*In vivo* imaging	Zebrafish	[111]
CV acetate, wax-like PEG sample, SiC powders	Red	520/620	*In vivo* imaging system	*In vivo* imaging of tumor	Tumor-bearing mice	[112]
Wheat straw and bamboo residues	Blue	420/–	CLSM	Imaging of cells	SP2/0	[113]
	Red	540/–	*In vivo* imaging system	*In vivo* imaging of tumor	Smmc-7721 tumor-bearing mice	
CA, H_3_PO_4_, EDA	Green	340/430	FM	Imaging of cells	RAW 264.7	[114]
	Red	450/500	*In vivo* imaging system	*In vivo* imaging of tumor	SGC7901 tumor-bearing BALB/c mice	

**Table 2:** Imaging-supported sensing applications using FL CDs.

Precursors/forms	FL color	Applied Ex/Em (nm)	Microscopic	Application	Biotarget	Ref.
Ascorbic acid, L-arginine	Green	750/380–495	Two-photon CLSM	Imaging of tissues	Pigskin tissue	[120]
	Red	750/500–650		Sensing of Fe3+	Fibroblast skin cells	
Abelmoschus manihot	Blue	330/410	FM	Sensing of 2,4,6-trinitrophenol (TNT)	Hela	[121]
Casein	Blue	383/446	CLSM	Sensing of Hg^2+^, biothiols	HeLa	[122]
Catechol, triethylene tetramine	Green	415/515	CLSM	Sensing of Fe^3+^, ascorbic acid (AA)	MCF-7	[123]
p-phenylenediamine, ammonia	Green	361/515	CLSM	Sensing of CrVI, TNT, and AA	SMMC7721	[124]
p-aminosalicylic acid, ethyleneglycol dimethacrylate	Green	390/520	FM	Sensing of Fe^3+^	BT474	[125]
Glycerol, DAMO	Blue	350/442	CLSM	Sensing of Fe^3+^	Zebrafish, Hela,	[126]
				Cancer/normal cell differentiation	A549, Hep G2/ AT II, L02	
Glutaraldehyde	Blue	440/–	CLSM	Sensing of microRNA-21	MCF-7	[127]
nitro benzaldehyde		360/–				
benzaldehyde		360/–				
CDs-chitosan						
White pepper, H2N-PEG-NH2	Green	420/525–550	CLSM	Sensing of coenzyme A	HeLa	[128]
	Red	420/>560				
CA, PEI	Blue	350/450	CLSM	Sensing of H_2_O_2_	HeLa	[129]
CQD-AuNC	Red	550/620				
CA, melamine	Blue	360/440	CLSM	Sensing of Hg^2+^, glutathione (GSH)	BHK	[130]
o-phenylenediamine	Green	488/–	CLSM	Sensing of atrazine	*E. coli, S. aureus*	[131]
2,3-diaminophenazine	Green	495/530	CLSM	Sensing of NAD^+^	A375 cells	[132]
Fungus fibers	Blue	360/440	FM	Sensing of tetracyclines	HepG2	[133]
CA, EDA	Blue	345/453	CLSM	Sensing of CA125	OVCAR-3	[134]
CD-aptamer						
CA, L-cysteine	Blue	355/425	FM	Sensing of testosterone	293T	[135]
*β*-CD-CDs						
L-tartaric acid, triethylenetetramine	Blue	350/425	CLSM	Sensing of metronidazole	MCF-7	[136]
CA	Blue	380/450	FM	Sensing of cathepsin B	HeLa	[137]
AS1411-Ce6-CQDs						
m-aminophenol	Yellow–green	450/520	CLSM	Sensing of selenol	L929	[138]
CD-DNS						
Food grade agave nectar, *α*-methoxy-*ω*-phosphate PEG	Red	430/600	*In vivo* imaging system	Imaging of hydroxyapatite-targeted bone	Athymic nude mice	[119]
CA, EDA	Blue, yellow	360/440, 565	CLSM	Sensing of thioredoxin reductase	MCF-7, HeLa cells	[139]
Biotin-CD-Naph						
Neutral red, triethylamine	Yellow	478/532, 618	CLSM	Sensing of Ag^+^, GSH	SMMC7721	[140]
Chestnut, onion	Blue	370/440	CLSM	Sensing of coenzyme A	T24	[141]
Aconitic acid, tryptophan	Blue	370/455	CLSM	Sensing of cytochrome c	HepG-2, zebrafish	[142]
FO-Pte, FO-PSe	Green	800/400–600	Two-photon CLSM	Sensing of superoxide anion	Hela, A549	[143]
					Breast tumor tissue	
EDTA-2Na, CuCl2	Blue	370/480	CLSM	Sensing of H_2_S	H3122	[144]
CA	Blue	405/470	CLSM	Sensing of Fe^3+^, AA	HepG2, zebrafish, liver ischemia tissue	[145]
CDs-DB	Red	405/450–550				
CA, phenosafranine,	Orange	525/600	CLSM	Sensing of nitrite	A549	[146]
HAuCl4, GSH, and glucose	Green	405/495–575	FM	Sensing of SKBR3 exosomes	HeLa	[147]
PEI-GCDs-Ab						
CA, 2,3-Phenazinediamine	Yellow	380/568	FM	Sensing of Ag^+^, GSH	H1299	[148]
CA, urea, and triethylenetetramine	Blue	380/470	CLSM	Sensing of Cu^2+^, GSH	Yeast	[116]
CA, methionine	Blue	350/420	FM	Sensing of Al^3+^	HUVEC	[149]
	Green	350/502				
Dunaliella salina	Green	340/415	FM	Imaging of cells	HEK-293	[150]
	Red			Sensing of Hg^2+^, Cr^6+^		
Alkali lignin, EDA, and formaldehyde	Blue	405/–	CLSM	Imaging of cells	RAW264.7	[151]
	Green	488/–		Sensing of Fe^3+^		
	Red	558/–				
Ocimum sanctum	Blue	330–385/–	FM	Imaging of cells	MDA-MB 468	[152]
	Green	450−480/–		Sensing of Pb^2+^		
	Red	510–550/–				
Banana plant	Blue	408/–	CLSM	Sensing of Fe^3+^	Hela, MCF-7	[153]
	Green	488/–				
	Red	561/–				
Ganoderma lucidum spores	Blue	405/–	CLSM	Sensing of Fe^3+^	MIHA	[154]
	Green	488/–				
	Red	559/–				
Phthalic acid, EDA, and H3PO4	Blue	405/422	CLSM	Imaging of cells	SMMC-7721	[155]
	Green	488/500		Sensing of Mn^7+^		
	Red	543/650				
Phthalocyanine	Green	780/520	Two-photon CLSM	Imaging of cells	MCF-7	[118]
	Red	850–890/600		Sensing of Fe^3+^		
Magnolia liliiflora	Blue	405/–	CLSM	Sensing of Fe^3+^	*Clone 9 hepatocytes*	[156]
	Green	488/–				
	Red	555/–				
Sweet potato	Blue	330–388/405	CLSM	Imaging of cells	Hela, HepG2	[157]
	Green	450–480/–		Sensing of Fe^3+^		
	Red	510–550/–				
Glucose, octadecylamine, and octadecene	Green	425/485	CLSM	Sensing of Cu^2+^	HepG2, HL-7702	[158]
HCD-based micelle	Red	425/655				
Syringa obtata Lindl	Blue	340/425	CLSM	Sensing of Fe^3+^	MCF-7	[159]
	Green	450/520				
Black soya beans	Blue	405/–	CLSM	Imaging of cells	SMMC-7721	[160]
	Green	488/–		Sensing of Fe^3+^		
	Red	543/–				
Aspartame	Blue	405/420–480	CLSM	Imaging of cells	SGC-7901	[161]
	Green	405/500–560		Sensing of Fe^3+^		
	Red	555/600–700				
o-phenylenediamine, 4,5-difluoro-1,2-benzenediamine, and tartaric acid	Green	480/600	FM	Imaging of cells	HEK 293T, NIH 3T3,	[162]
	Red	540/550		Sensing of Ag^+^	COS-7, HepG2, and B16F10	
Aminosalicylic acid	Green	405/–	CLSM	Sensing of Fe^3+^	H1299	[163]
	Yellow	488/–				
	Red	542/–				
CA, thiourea	Blue	405/450	FM	Imaging of cells	MiaPaCa-2	[164]
				Sensing of Fe^3+^		
L-glutamic acid, EDA	Blue	360/459	CLSM	Imaging of fungi	*C. gloeosporioides*	[165]
				Sensing of Fe^3+^		
m-phenylenediamine, diethylenetriaminepenta (methylenephosphonic acid)	Green	440/510	CLSM	Imaging of cells	A549, KB	[166]
				Sensing of Fe^3+^		
CA, diethylenetriamine	Blue	391/438	FM	Sensing of Co^2+^	HeLa	[167]
Osmanthus fragrans	Blue	340/410	FM	Sensing of Fe^3+^, AA	A549	[168]
CA, methylamine hydrochloride, and lanthanum	Green	420/510	FM	Sensing of Fe^3+^	HeLa	[169]
chloride heptahydrate						
Tetraphenylporphyrin-Mn, CA	Blue	330–385/–	FM	Sensing of Fe^3+^	HeLa, zebrafish	[170]
	Green	400–440/–				
	Red	510–550/–				
P-phenylenediamine	Orange	566/590	CLSM	Sensing of intracellular pH	SMMC7721	[171]
CA, 1,4-butanediamine	Blue	380/443	CLSM	Sensing of intracellular pH	*Pholiota adipose fungi*	[172]
RhB-AB-CDs	Red	400/580				
p-phenylenediamine	Red	488/550–650	CLSM	Imaging of cells	HepG2, HL-7702	[173]
				Sensing of intracellular polarity		
Ascorbic acid	Yellow	405/415–550	CLSM	Imaging of nucleolus	293T	[174]
				Sensing of temperature		

**Table 3:** : Imaging-guided therapeutic applications using FL CDs.

Precursors/Forms	FL color	Applied Ex/Em (nm)	Microscopic	Application	Biotarget	Ref.
Bamboo leaves CDs-CBBA-Dox	Green	488/–	CLSM	Imaging of cells Imaging-guided chemotherapy	HeLa	[86]
*Hypocrella bambusae*	Red	540/610	CLSM	Imaging of cells	Hela	[175]
			*In vivo* imaging system	Imaging-guided PDT/PTT	4T1 tumor-bearing mice	
CA, hyaluronic acid, and PEI	Blue	341/461	CLSM	Imaging of cells	4T1	[176]
CD@p-CBA-DOX			*In vivo* imaging system	Imaging-guided CD44-targeted chemotherapy	4T1 tumor-bearing BALB/c mice	
Dopamine hydrochloride, folic acid	Blue	425/485	FM	Imaging-guided PTT	LNCaP	[177]
4-amino salicylic acid	Yellow	490/547	FM	Imaging of cells	MCF-7/ADR	[178]
			*In vivo* imaging system	Imaging-guided chemotherapy	MCF-7/ADR tumor-bearing mice	
CA, EDA, hyaluronic acid	Blue	405/–	CLSM	Imaging-guided chemotherapy	A549 tumor-bearing mice	[179]
MSN-SS-CD_HA_-Dox	Green	488/–	*In/Ex vivo* imaging system			
	Red	561/–				
CA, Ru-Aphen	Red	490/616	CLSM	*In vivo* imaging	Zebrafish	[180]
				Imaging-guided PDT	HeLa	
1,3,6-trinitropyrene	Green	457/570	CLSM	Imaging of lysosome-targeted cells	HeLa	[181]
			*In vivo* imaging system	Imaging-guided PDT, PTT	4T1-tumor-bearing nude mice	
CA, folic acid, DOX	Blue	405/488	CLSM	Imaging of cells	HepG2	[182]
				Imaging-guided chemotherapy	Liver cancer	
L-cysteine, EDA, and Ru(II) complex	Red	405/660	Two-photon	Imaging of lysosome-targeted cells	A549	[117]
		810/660	CLSM	Imaging-guided PDT	Zebrafish	
hydroxyapatite NPs	Green	455/–	*In vivo* imaging system	Imaging-guided chemotherapy	Tumor-bearing mice	[183]
C-hMOS-Dox	Red	523/–				
CA, HPAP	Blue	405/–	*In vivo* imaging system	Imaging-guided gene therapy	MCF-7 tumor-bearing BALB/c	[184]
PPD@HPAP-CDs/pDNA	Green	488/–			nude mice	
	Red	543/–				
Sodium citrate, ammonium	Blue	350/435	FM	Imaging of cells	A549	[185]
				Imaging-guided chemotherapy		
Bicarbonate CDs/Dox/ G5–RGD–TPGS						
6-O-((O,O'-Di-lauroyl)tartaryl)-d-glucose, WS_2_@CDs	Cyan	405/445	CLSM	Imaging of cells	HeLa	[186]
	Green	440/477		Imaging-guided PTT		
	Red	568/640				
4-aminophenol	Red	540/620	*In vivo* imaging system	Imaging-guided chemotherapy	Hela tumor-bearing mice	[187]
CSCNP-R-CQDs/Dox						
Watermelon juice	Blue	360/–	*In vivo* imaging system	NIR-II FL imaging-guided PTT	Hela tumor-bearing BALB/C mice	[188]
	NIR-II	808/925				
F127-mPR, formalin, and phenol	Blue	405/–	CLSM	Imaging of cells	U87	[189]
	Green	458/–	*In vivo* imaging system	Imaging-guided PTT	Glioma-bearing mice	
	Yellow	488/–				
	Red	514/–				
CA, PEI	Red	550/640	CLSM	Imaging of cells	MCF-7, HeLa, and 4T1	[190]
CD-Ce6			*In vivo* imaging system	Imaging-guided PDT/PTT	4T1 tumor-bearing BALB/c mice	
CA, GdCl3, poly-lysine	Blue	350/450	CLSM	Imaging of cells	Hela	[191]
FA-GdN@CQDs-MWCNTs			*In vivo* imaging system	Imaging-guided chemo/PTT	HeLa tumor-bearing mice	
Manganese(II) phthalocyanine	Red	690/745	CLSM	Imaging of cells	Hela	[192]
			*In vivo* imaging system	Imaging-guided PDT	4T1 tumor-bearing mice	
Pheophytin powder	Red	620/680	CLSM	Imaging of cells	4T1	[193]
			*In vivo* imaging system	Imaging-guided PDT	4T1 tumor-bearing mice	
CA, formamide	Red	620/650	CLSM	Imaging of cells	MCF-7	[194]
HFn(DOX)/CDs			*In vivo* imaging system	Imaging-guided chemo/PDT	S180 tumor-bearing mice	
CA	Red	633/640/750	CLSM	Imaging of cells	4T1	[195]
CyOH–AgNP/CD			*In vivo* imaging system	Imaging-guided PDT	4T1 tumor-bearing mice	
Polythiophene	Red	635/690	CLSM	Imaging of cells	HeLa	[196]
CDs/MnO2-PEG			*In vivo* imaging system	Imaging-guided PDT	4T1-luc tumor-bearing mice	
Polythiophene, diphenyl diselenide	Red	500/730, 820	Two-photon	Imaging of cells	HeLa	[197]
			CLSM	Imaging-guided PTT	4T1 tumor-bearing mice	
			*In vivo* imaging system			
